The article "Protein tyrosine phosphatase receptor type Z1 inhibits the cisplatin resistance of ovarian cancer by regulating PI3K/AKT/mTOR signal pathway" was retracted in 2024. Reasons: original data or images not available; concerns about the data; concerns about the results or conclusions.

# Protein tyrosine phosphatase receptor type Z1 inhibits the cisplatin resistance of ovarian cancer by regulating PI3K/AKT/mTOR signal pathway

**DOI:** 10.1080/21655979.2021.2022268

**Published:** 2022-01-09

**Authors:** Peng Wang, Yuanjing Hu, Pengpeng Qu, Ying Zhao, Jing Liu, Jianguo Zhao, Beihua Kong

**Affiliations:** a Department of Gynecology Oncology, Qilu Hospital, Cheeloo College of Medicine, Shandong University, Jinan, Shandong, China; b Department of Gynecology Oncology, Tianjin Central Hospital of Obstetrics and Gynecology, Tianjin, China

**Keywords:** Ovarian cancer, PTPRZ1, cisplatin, PI3K/AKT/mTOR

## Abstract

Most patients with ovarian cancer (OC) get remission after undergoing cytoreductive surgery and platinum-based standard chemotherapy, but more than 50% of patients with advanced OC relapse within the first 5 years after treatment and develop resistance to standard chemotherapy. The production of medicinal properties is the main reason for the poor prognosis and high mortality of OC patients. Cisplatin (DDP) resistance is a major cause for poor prognosis of OC patients. PTPRZ1 can regulate the growth and apoptosis of ovarian cancer cells, while the molecular mechanism remains unknown. This study was designed to investigate the roles of PTPRZ1 in DDP-resistant OC cells and possible mechanism. PTPRZ1 expression in OC tissues and normal tissues was analyzed by GEPIA database and verified by Real-time Quantitative Reverse Transcription PCR (RT-PCR) assay. PTPRZ1 expression in normal ovarian cancer cells and DDP-resistant OC cells was also analyzed. Subsequently, RT-PCR, Western blot, MTT experiment and flow cytometry were used to assess the effects of PTPRZ1-PI3K/AKT/mTOR regulating axis on DDP resistance of OC. PTPRZ1 expression was abnormally low in OC tissues, and notably reduced in DDP-resistant OC cells. MTT experiment and flow cytometer indicated that overexpression of PTPRZ1 enhanced the DDP sensitivity of OC cells and promoted the cell apoptosis. Moreover, the results of our research showed that PTPRZ1 might exert its biological effects through blocking PI3K/AKT/mTOR pathway. PTPRZ1 overexpression inhibitied OC tumor growth and resistance to DDP in vivo. Overall, PTPRZ1 might suppress the DDP resistance of OC and induce the cytotoxicity by blocking PI3K/AKT/mTOR pathway.

## Introduction

Ovarian cancer (OC) is a leading death cause of all gynecological malignant tumors, while epithelial ovarian cancer (EOC) is the most common OC [1]. With the development of laparoscopic surgery, robot assisted surgery and adjuvant chemotherapy for OC, the perioperative effects and prognosis of some OC patients are improved. Moreover, The 10-year survival rate of patients diagnosed with advanced-stage OC is 15%, compared with 55% for those diagnosed with early-stage disease [2]. The late diagnosis of OC is normally because the cancer is asymptomatic as it lies deep in the abdomen. Therefore, the cancer is presented late and manifest as advanced stage and requires chemotherapy. However, as a result of toxic and side effects and drug resistance of chemotherapeutic drugs, the chemoresistance, tumor recurrence, extensive metastasis occur in most cases, and finally result in patient death [3,4]. Hence, it is imminent to find the key molecules and potential molecular mechanisms that may cause ovarian cancer to resist DDP.

The fist-line therapeutic regimens of OC include complete cytoreductive surgery and platinum- (cisplatin or carboplatin) and taxane-(paclitaxel)-based first-line combined chemotherapy [5–7]. Many patients, especially uncontrolled or early recurrence patients, are vulnerable to progression into platinum resistance, thereby affecting their survival [8,9]. Therefore, platinum resistance has become an obstacle for chemotherapy and an important clinical challenge. Until now, there are very limited measures to prevent or reverse platinum resistance.

PTPRZ1 is mainly expressed in central nervous system, identified as a key factor for the recovery of demyelination damage, and is abnormally expressed in multiple tumors recently. For instance, PTPRZ1 is considered as an oncogene for promoting tumor growth in glioma that further results in the malignant progression of glioma by fusion with MET proto-oncogene, receptor tyrosine kinase (MET) [10]; in breast cancer, PTPRZ1 reduces the chemosensitivity through promoting tumor cell growth and suppressing cell apoptosis [11]; the proliferation of renal cell carcinoma (RCC) cells enhanced by PTPRZ1 is dependent on the inactivation of von Hippel-Lindau tumor suppressor (VHL), while PTPRZ1/β-catenin pathway may be a potential target for the treatment of non-active VHL RCC [12].

We observed that PTPRZ1 expression was considerably reduced in OC through bioinformatic analysis and RT-PCR detection. Meanwhile, further detection revealed that its expression in DDP resistant cell lines was lower than that in normal cell lines. Therefore, with this point, we initially explored the roles of PTPRZ1 in DDP resistance of OC and their possible mechanism to provide new thoughts for clinical diagnosis and treatment of OC.

## Method

### GEPIA database

The expression of mRNA profile was analyzed in 426 OC tissues and 88 normal control tissues obtained from The Cancer Genome Atlas (TCGA) database. GEPIA is a new interactive website for the analysis of RNA sequence data based on TCGA and GTEx (http://gepiacancer-pku.cn/index.html) [13]. PTPRZ1 expression in OC tissues and normal control tissues was analyzed. The association of PTPRZ1 expression with the overall survival (OS) and disease free survival (DFS) of OC patients was calculated by GEPIA database.

### Sample collection

Thirty pairs of OC tissues and normal control tissues were collected from Qilu Hospital and Tianjin Central Hospital of Obstetrics and Gynecology. All OC patients received no chemotherapy or radiotherapy before surgery. In addition, a total of 20 patients with OC who underwent radical surgery and received the same DDP-based combination chemotherapeutic regimen at Qilu Hospital, Shandong University were retrospectively collected. We defined chemo-resistance or chemo-sensitivity as a relapse/progression within 6 months or after 6 months from the ending day of last platinum-based chemotherapy, respectively. Pathological classification and tumor staging were conducted according to the cancer staging criteria of Union for International Cancer Control. This study protocol was approved by the ethics committee of Qilu Hospital and Tianjin Central Hospital of Obstetrics and Gynecology. All patients signed the informed consent. This study was performed following the Declaration of Helsinki.

### Cell culture

Ovarian cancer cell lines SKOV3 and A2780 were commercially acquired from the Shanghai Institute of Biochemistry and Cell Biology, CAS (Shanghai, China). Cells were cultured in Dulbecco modified Eagle’s culture medium containing 10% fetal bovine serum (Gibco, Carlsbad, California) in an incubator with 5% carbon dioxide at 37°C. Drug-resistant cell lines SKOV3 and A2780 were constructed by treating the proliferated cell cultures using DDP (Meilun Biotech, Dalian, China) at a concentration of 8 μM for consecutive 12 weeks [14].

### Cell transfection

A total of 5 × 10^4^/ml SKOV3 and A2780 cells (or SKOV3/DDP and A2780/DDP) were seeded into 6-well plate, and the transfection was performed at a cell density of about 70% by reference to the instructions for use of Lipofectamine 3000 (Invitrogen, USA) [15]. Cells were transfected by using PTPRZ1 overexpression plasmids and corresponding negative references. Above transfection reagents and corresponding negative references were designed and synthesized by GenePharma (Shanghai, China). Cells were collected for subsequent experiments after 48 h of transfection.

### Real-time Quantitative Reverse Transcription PCR (RT-PCR) assay

All the OC tissues and cell lines were extracted by using TRIzol reagent (Invitrogen, CA, USA) as per the instructions for use [16]. Post chloroform extraction, the aqueous phase was transferred into a new tube. Isopropanol was used to subside RNAs in the aqueous phase. RNA sediments were washed by using 75% ethyl alcohol and dried at room temperature. DEPC water was then added for resuspension. RNAs were subject to reverse transcription into cDNAs by using PrimeScript RT reagent Kit (TAKARA, Code No. RR036A) according to its instructions for use. For RT-PCR, SYBR® Green Master Mix (TaKaRa) was used for the detection on Roche480 as per the instructions for use. GAPDH was used as the internal reference, and the calculation was performed with 2^−ΔΔCT^ method [17]. The primer sequence is presented below: PTPRZ1 forward: GCCTGGATTGGGCTAATGGAT, PTPRZ1 reverse: CAGTGCTCCTGTATAGGACCA; GAPDH forward: GGAGCGAGATCCCTCCAAAAT, GAPDH reverse: GGCTGTTGTCATACTTCTCATGG.

### MTT experiment

MTT experiment was conducted based on the previous research [18]. Cells were seeded into the 96-well plate at 4 × 10^3^ cells per well. DDP at the concentration of 0 μM, 1 μM, 2 μM, 5 μM, 10 μM, 20 μM and 40 μM was added into each group. The plate was then incubated for 48 h at 37°C. Subsequently, the culture solution was replaced with new culture medium. With MTT (0.5 mg/ml) added, the plate was incubated with 5% CO_2_ at 37°C for 4 h. The culture solution was then carefully removed, and 150 μl DMSO was added into each well to fully dissolve the generated formazan crystals. The microplate reader was used for absorbance measurement at the wavelength of 570 nm. The experiment was repeated in triplicate.

### Cell apoptosis experiment

Cell apoptosis experiment was conducted based on the previous research [19]. After cell transfection, with SKOV3/DDP and A2780/DDP cells collected and washed with PBS, cells were stained by using Annexin V-FITC kit (Beyotime, China) according to the instructions for use. FACSCalibur Flow Cytometer (BD Bioscience, Franklin Lakes, NJ, USA) was then utilized to analyze the cell apoptosis rate.

### Western blot

Western blot experiment was conducted based on the previous research [20].Transfected SKOV3/DDP and A2780/DDP cells were collected. Upon protein extraction, cell lysis solution containing protease inhibitor PMSF (Beyotime, Nantong, China) was added. On the ice, the supernatant was collected post centrifugation. The protein concentration was detected by using BCA Protein Quantitation Kit (Beyotime, Nantong, China) as per its operating instructions. For albuminous degeneration, cells were heated at 100°C after adding SDS-PAGE protein loading buffer. The transfer membrane was conducted after the loading buffer was used up. Corresponding size of PVDF membrane cut as per the molecular weight was subject to antigen blocking in 5% skim milk powder blocking buffer. The incubation was conducted by adding primary antibodies. Another incubation was then performed by using secondary antibodies for subsequent exposure.

### Animal studies

The animal studies were conducted according to the institutional ethics guidelines for animal assays approved by the animal management committee of Shandong University. About 5 × 10^6^ cells were injected subcutaneously into the axilla of the female athymic BALB/C nude mice. After 1 week, mice were then randomized into two groups and treated with DDP (5 mg/kg) or normal saline (NS) weekly. The tumor volume was calculated using the following formula: volume (mm^3^) = length × width^2^ /2 [21]. Every group was treated by 6 cycles of DDP/NS treatment until mice were euthanized, and tumors were removed for further study.

### Data analysis

The data were analyzed with SPSS 20.0 and GraphPad Prism 6.0 statistical software. The measurement data were shown as the mean ± standard deviation. Two sample t-test was used as the statistical method for between-group comparison. P < 0.05 was considered statistically significant.

## Results

In this sutudy, we found that PTPRZ1 expression was abnormally low in OC tissues, and notably reduced in DDP-resistant OC cells. *In vitro* experiments indicated that overexpression of PTPRZ1 could enhance the DDP sensitivity of OC cells and promoted the cell apoptosis. Moreover, the results of our research demonstrated that PTPRZ1 might exert its biological effects by blocking PI3K/AKT/mTOR pathway.

### PTPRZ1 expression was reduced in OC

The analysis of OC tissues and normal control tissues through GEPIA database found that PTPRZ1 expression was reduced in OC tissues (Figure 1a). The correlation of PTPRZ1 expression with OS and DFS of OC patients was then analyzed via TCGA database, which showed no significant correlation between PTPRZ1 and OS or DFS (Figure 1b,c). Subsequently, RT-PCR was conducted for PTPRZ1 expression in 30 OC tissues and 30 control tissues and revealed significant reduction of PTPRZ1 expression in OC tissues (Figure 1d). We also found that PTPRZ1 was downregulated in DDP-resistant OC tissues compared with DDP-sensitive OC tissues (Figure 1e). Moreover, PTPRZ1 expression in DDP-resistant OC tissues SKOV3/DDP and A2780/DDP was significantly lower than that in normal OC cells (figure 1f).

**Figure 1.** PTPRZ1 expression was reduced in OC. (a) PTPRZ1 expression in OC tissues and normal control tissues as analyzed by GEPIA database. (b) The analysis of TCGA database uncovered no considerable association of PTPRZ1 expression with OS of OC patients. (c) The analysis of TCGA database revealed no remarkable correlation of PTPRZ1 expression with DFS of OC patients. (d) Relative expression of PTPRZ1 in OC tissues and normal control tissues by RT-PCR. (e) Relative expression of PTPRZ1 in DDP-sensitive OC tissues and DDP-resistant OC tissues by RT-PCR. (f) Lower PTPRZ1 expression in DDP-resistant OC cells relative to normal OC cells.

Data was expressed as mean ± SD. *p < 0.05.

### PTPRZ1 overexpression made OC cells sensitive to cisplatin-induced cytotoxicity

PTPRZ1 expression was increased by overexpression plasmids in OC cells SKOV3 and A2780, and transfection efficiency was detected through RT-PCR (Figure 2a). Subsequently, different concentrations of cisplatin were used to treat the transfected cells. The results suggested that PTPRZ1 overexpression made OC cells sensitive to cisplatin-induced cytotoxicity (Figure 2b). The analysis revealed that PTPRZ1 overexpression could considerably reduce the half-maximal inhibitory concentration (IC50) of cisplatin for OC (Figure 2c).

**Figure 2.** PTPRZ1 overexpression made OC cells sensitive to cisplatin-induced cytotoxicity. (a) Transfection efficiency of PTPRZ1 overexpression plasmids in OC cells SKOV3 and A2780 by RT-PCR. (b) The cytotoxicity of different concentrations of cisplatin was increased in cells lines SKOV3 and A2780 by transfection with PTPRZ1 overexpression plasmids. (c) Effects of PTPRZ1 on IC50 of cisplatin in cell lines SKOV3 and A2780. Data was expressed as mean ± SD. *p < 0.05; ***p < 0.001.

### PTPRZ1 negatively regulated DDP sensitivity of OC cells

The biological effects of PTPRZ1 were further verified in DDP-resistant OC cells SKOV3/DDP and A2780/DDP. Similarly, PTPRZ1 expression in cells was firstly increased with PTPRZ1 overexpressed plasmids (Figure 3a). After transfected SKOV3/DDP and A2780/DDP cells were treated with different concentrations of cisplatin, MTT experiment uncovered that the transfection with oe-PTPRZ1 in cells enhanced the cisplatin sensitivity of cells (Figure 3b) and reduced the IC50 of cisplatin for OC relative to the control group (Figure 3c).

**Figure 3.** PTPRZ1 negatively regulated DDP sensitivity of OC cells. (a) Transfection efficiency of PTPRZ1 overexpression plasmids in DDP-resistant OC cells SKOV3/DDP and A2780/DDP by RT-PCR. (b) The cytotoxicity of different concentrations of cisplatin was enhanced in cell lines SKOV3/DDP and A2780/DDP by transfection with PTPRZ1 overexpression plasmids. (c) Effects of PTPRZ1 on IC50 of cisplatin in cell lines SKOV3/DDP and A2780/DDP. Data was expressed as mean ± SD. *p < 0.05; **p < 0.01; ***p < 0.001.

### PTPRZ1 overexpression suppressed PI3K/AKT/mTOR pathway

After transfection with oe-NC and oe-PTPRZ1 in DDP-resistant OC cells SKOV3/DDP and A2780/DDP, respectively, the phosphorylation level of AKT and mTOR proteins was detected by Western blot. The results revealed that PTPRZ1 overexpression in SKOV3/DDP and A2780/DDP cells could decrease p-AKT and p-mTOR protein expression. Additionally, PTPRZ1 exerted its biological effects by suppressing PI3K/AKT/mTOR pathway (Figure 4).

**Figure 4.** PTPRZ1 regulated PI3K/AKT/mTOR pathway in cell lines SKOV3/DDP and A2780/DDP. Phosphorylation level of AKT and mTOR detected by Western blot experiment post overexpression of PTPRZ1 in cell lines SKOV3/DDP and A2780/DDP. Data was expressed as mean ± SD. **p < 0.01.

### The activation of PI3K/AKT/mTOR pathway reversed PTPRZ1 overexpression mediated pro-apoptotic effects

To further verify whether PTPRZ1 involved in the cisplatin resistance process of OC via regulating PI3K/AKT/mTOR pathway, with PTPRZ1 overexpression and transfection with PI3K/AKT/mTOR agonist IGF-1 in SKOV3/DDP and A2780/DDP cells, cell apoptosis was detected using a flow cytometer. In Figure 5a, after PTPRZ1 was overexpressed in SKOV3/DDP and A2780/DDP cells, notably higher proportion of cell apoptosis was observed; this proportion was reduced post transfection with IGF-1. Furthermore, PTPRZ1 overexpression enhanced the protein level of C caspase and BAX and suppressed the protein level of BCL-2; with concurrent transfection with IGF-1, lower protein level of C caspase and BAX and higher protein level of BCL-2 were observed (Figure 5b). These findings objectivized that PTPRZ1 regulated the chemosensitivity of cisplatin to OC cells by regulating PI3K/AKT/mTOR pathway.

**Figure 5.** The activation of PI3K/AKT/mTOR pathway reversed PTPRZ1 overexpression mediated pro-apoptotic effects. (a).Apoptosis of SKOV3/DDP and A2780/DDP cells post treatment with PTPRZ1 overexpression plasmids and PI3K/AKT/mTOR agonist IGF-1 by flow cytometry. (b) Protein level of C caspase, BAX and BCL-2 in SKOV3/DDP and A2780/DDP cells post treatment with PTPRZ1 overexpression plasmids and PI3K/AKT/mTOR agonist IGF-1 by Western blot experiment. Data was expressed as mean ± SD. **p < 0.01; ***p < 0.001, # *p* < 0.05; ## *p* < 0.01.

### *PTPRZ1 overexpression inhibitied OC tumor growth and resistance to DDP* in vivo

Furthermore, we established stably expressed PTPRZ1 (LV-PTPRZ1) SKOV3/DDP cells and the corresponding control cells to treat immunodeficient mice. The mice were sacrificed and analyzed after 4 weeks. The results showed that LV-PTPRZ1 reduced tumor growth and resistance to DDP *in vivo* compared with LV-NC (Figure 6a–c).

**Figure 6.** PTPRZ1 overexpression inhibitied OC tumor growth and resistance to DDP in vivo. (a) Typical images of tumors from LV-NC/DDP group and LV-PTPRZ1/DDP group of nude mice. (b) Measurement of tumor volumes. (c) Measurement of tumor weight.

Data was expressed as mean ± SD. *p < 0.05.

## Discussion

OC is susceptible to difficult early diagnosis, chemoresistance, and recurrence, with 5-year survival rate of only about 40%, thus it has been a hotspot among clinicians [22]. Main causes for low survival rate of OC include low early diagnosis and susceptibility to recurrence or metastasis. Previous studies showed that in addition to unique characteristics of OC, less sensitivity of OC cells to chemotherapeutic drugs was also a cause for recurrence, metastasis and then failure of tumor treatment [23,24]. Since targeted therapy is a means for tumor treatment by selective inhibition of molecular pathway, a question is raised that whether selective targeted therapy may be provided for the resistance mechanism. At present, there is no available clinical trial to demonstrate the ideal response rate of targeted therapy. Neither single-target therapy nor combination with current chemotherapy regimens improves the drug resistance or significantly increase the patients’ survival rate.

Early bioinformatic analysis and RT-PCR detection revealed notably low expression of PTPRZ1 in OC. For this reason, we made further study. The reason why cisplatin was selected as the study subject for drug resistance was that platinum drugs had become indispensable drugs for OC chemotherapy. It exerted cytotoxic effects in cells and had chemotherapy effects. The specific mechanism preliminarily confirmed a possible association with apoptosis process [25,26]. Cisplatin is the first-line chemotherapeutic drug for OC, and there is a close association of platinum resistance with postoperative survival of OC patients [27,28]. PTPRZ1 expression was considerably reduced in DDP-resistant OC cell lines as detected. In vitro cell experiments suggested that PTPRZ1 overexpression made OC cells sensitive to cisplatin-induced cytotoxicity and considerably reduced the IC50 of OC for cisplatin.

Previous studies have shown that the PI3K-AKT pathway plays an important role in DDP resistance [29–32]. We speculate dwhether PTPRZ1 was involved in DDP resistance of OC by regulating the PI3K-AKT pathway. In Western blot, overexpression of PTPRZ1 suppressed the phosphorylation level of AKT and mTOR, suggesting that PTPRZ1 participated in the cisplatin resistance of OC possibly through inhibiting PI3K/AKT/mTOR pathway. PI3K/AKT/mTOR pathway is a signal transduction pathway extensively distributed in cells to involve in cell growth, suppress cell apoptosis and maintain important functions of cells [33,34]. P13 K may be activated by multiples factors including insulin-like growth factor (IGF-1) to activate the downstream AKT via phosphorylation. Activated AKT may phosphorylate tuberous sclerosis complex 2 and attenuate the inhibiting effect of TSC2 on its downstream mTOR [35–37]. MTOR is an intracellular serine-threonine kinase that is highly conservative for its evolution. It is widely expressed in various biological cells. The activation of mTOR phosphorylates the downstream P70S6K1 effector to initiate the translation process and promote the synthesis of RNA and proteins [38,39]. This pathway participates in the occurrence and development of multiple tumors and angiogenesis, and is also considered as the primary pathway for cancer cell survival [40,41]. Then, in vitro cell experiment indicated that the transfection with PI3K/AKT/mTOR pathway agonist IGF-1 recovered the pro-apoptotic effects of PTPRZ1 overexpression.

Meanwhile, this study also had many limitations. Firstly, other downstream targets of PTPRZ1 should be explored and verified in future studies. Furthermore, the correlation between the expression level of PTPRZ1 and the clinical characteristics of patients with OC needs to be further explored. Moreover, The results of the TCGA database showed that the expression level of PTPRZ1 was not significantly correlated with OS and DFS in OC patients. We suspect that the expression level of PTPRZ1 may be related to the prognosis of DDP sensitivity and resistance patients. However, there are few specimens collected at present, and we will explore this issue in further research. In future studies, we will collect more clinical specimens and analyze the correlation between the expression level of PTPRZ1 and the clinical characteristics of OC patients. In addition, we will perform high-throughput sequencing analysis after knocking out PTPRZ1 in OC cells to explore the possible molecular mechanism of PTPRZ1 in OC. Taken together, this study initially confirmed that PTPRZ1 suppressed the cisplatin resistance of OC and induced the cytotoxicity by blocking PI3K/AKT/mTOR pathway. This provides new perspective and theoretical basis for clinical treatment of OC.

## Conclusion

Collectively, our present outcomes indicated that PTPRZ1 might enhance the DDP sensitivity of OC cells and promote the cell apoptosis by blocking PI3K/AKT/mTOR pathway, thereby improving the efficacy of DDP clinical treatment of OC.

## Data Availability

The datasets used and/or analyzed during the present study are available from the corresponding author on reasonable request.
